The article "Frequencies of Porphyromonas gingivalis Detection in Oral-Digestive Tract Tumors" was retracted in 2023. Reasons: unreliable results or conclusions; concerns about the data.

# Frequencies of *Porphyromonas gingivalis* Detection in Oral-Digestive Tract Tumors

**DOI:** 10.3389/pore.2021.628942

**Published:** 2021-04-01

**Authors:** Jinyu Kong, Xiang Yuan, Jian Wang, Yiwen Liu, Wei Sun, Bianli Gu, Zijun Lan, Shegan Gao

**Affiliations:** ^1^ Henan Key Laboratory of Cancer Epigenetics, Cancer Institute, The First Affiliated Hospital, College of Clinical Medicine of Henan University of Science and Technology, Luoyang, China; ^2^ Radiodiagnosis Center, The First Affiliated Hospital, College of Clinical Medicine of Henan University of Science and Technology, Luoyang, China

**Keywords:** *Porphyromonas gingivalis*, oral squamous cell carcinoma, oesophageal squamous cell carcinoma, digestive tract cancer, prognosis

## Abstract

Mounting evidence suggests a causal relationship between specific bacterial infections and the development of certain malignancies. In this study, we examined the presence of *Porphyromonas gingivalis* (*P. gingivalis*) in oral-digestive tract tumors by immunohistochemistry (IHC) and PCR and analyzed the correlation between *P. gingivalis* detection and clinicopathological characteristics and prognosis of oral and esophageal carcinoma. The IHC results showed that the positive rates of *P. gingivalis* were 60.00, 46.00, 20.00, 6.67, and 2.86% in oral, esophagus, cardiac, stomach, and colorectal cancer tissues, respectively. Likewise, PCR results showed rates of 56.00, 42.00, 16.67, 3.33, and 2.86%, respectively. The two methods were consistent, and the *kappa* value was 0.806, *P* < 0.001. In addition, *P. gingivalis* expression was significantly correlated with lymph node metastasis and the clinical stages of oral and esophageal cancer (*P* < 0.05). The overall survival rate of the *P. gingivalis* undetected group (86, 50%) was significantly higher than that of the *P. gingivalis* detected group (57, 14%) for oral and esophageal cancer, respectively. In conclusion, the detection rate of *P. gingivalis* showed a decreasing trend in oral-digestive tract tumors. Detection with *P. gingivalis* was associated with poor prognosis for oral and esophageal cancer.

## Introduction

The digestive tract consists of the oral cavity, pharynx, esophagus, stomach, and intestines. Digestive tract cancers are among the most common malignancies in the world [1]. Numerous epidemiological studies have demonstrated that lifestyle factors are associated with digestive tract cancers, such as smoking, alcohol intake, obesity, being underweight, and low consumption of vegetables and fruits [2]. In addition, chronic inflammation is widely considered to be a cause of digestive tract cancer, and a growing number of studies have revealed that approximately 20% of the morbidity and death of patients with cancer involve chronic inflammation induced by infectious agents [3]such as *Helicobacter pylori* in gastric cancer (GC) [4], *Prevotella melanin* in oral carcinomas [5], and *Fusobacterium nucleatum* in colorectal cancer (CRC) [6].

Epidemiological studies have demonstrated that periodontal diseases are significantly associated with upper digestive tract cancers and may even relate to survival [7]. *Porphyromonas gingivalis*, a Gram-negative anaerobic bacterium, is one of the most virulent bacteria in periodontal disease [8], and the relationship between *P. gingivalis* and oral and upper digestive tract tumors has attracted increasing attention. Oral and maxillofacial vein valves are few or absent, and blood is supplied abundantly, so pathogenic bacteria can easily circulate throughout the whole body [9]. An increasing number of studies have confirmed that *P. gingivalis* is strongly associated with the development of oral squamous cell carcinoma cancer (OSCC) [10], pancreatic cancers [11].

Although *P. gingivalis* has been proven to invade gingival epithelial cells [12], studies on its presence in the epithelium of different sites of the digestive tract are scarce. Previously, our group found that *P. gingivalis* detection may be a high-risk factor for esophageal squamous cell carcinoma (ESCC), and was correlated with the development of esophageal cancer [13–17]. These reports indicate that chronic bacterial infection with *P. gingivalis* is an important etiological factor of tumor development and progression. In addition, we also reported the occurrence of *P. gingivali*s in surgical specimens of the upper digestive tract. However, few studies have examined the presence of *P. gingivalis* in cardia and stomach tissue samples, and no studies have focused on *P. gingivalis* in colorectal cancer tissues. Therefore, the purpose of the present study was to detect the frequency of *P. gingivalis* in oral-digestive tract cancers including oral, esophagus, cardia, stomach and colorectal cancer tissues by IHC and PCR and to analyze the correlation between *P. gingivalis* and the prognosis of oral and esophageal carcinoma.

## Methods

### Patients and Human Tissues

This study was a retrospective analysis. Patients diagnosed with histologically confirmed primary tumors were recruited for this study, including 50 cases of OSCC, 50 cases of ESCC, 30 cases of gastric cardia adenocarcinoma (GCA), 30 cases of GC, and 35 cases of CRC at the First Affiliated Hospital of Henan University of Science and Technology during January 2012 through December 2018. Demographics (sex, age, smoking status, drinking status) and clinical information (differentiation status, lymph node metastasis, clinical stage) were collected from medical records (see Supplementary Table S1). The patients were followed up by outpatient service and telephone, and the end date of follow-up was 15 August 2018. The deaths of patients were 14 and 33 in OSCC and ESCC samples, respectively. One case of OSCC and two cases of ESCC were lost to follow-up, a loss rate of 2.00 and 4.00%, respectively. Overall survival (OS) was defined as the period from tumor diagnosis to the last follow-up or death from any cause.

The tumor specimens were taken from primary lesions, and then parts of them were frozen in liquid nitrogen at −80°C. Some portions were fixed by formaldehyde and embedded in paraffin. This study was approved by the Institutional Review Board of the University of Henan University of Science and Technology on July 23, 2018 (NO. 2018-03-B003). Each study participant signed an informed consent form, and they did not receive chemoradiotherapy or immunotherapy before surgery.

### Immunohistochemistry (IHC)

The cancer tissues were fixed in 10% formalin and then embedded in paraffin. Serial sections of 3 μm thickness were prepared and deparaffinized by submersion in xylene and four separate concentrations of ethanol (100, 95, 85, and 75%), and rinsing continuously in distilled water for 2 min. Antigen retrieval was performed by incubating the slides in 0.01 moL·L^−1^ citrate buffer (C1032, Solarbio, Beijing, China), and SP-9000 SPlink Detection Kit (Biotin-Streptavidin HRP Detection Systems, SP-9000, ZSGB-BIO, China) was used according to the manufacturer’s instructions. Polyclonal rabbit anti-*P. gingivalis* 33,277 (A gift from the University of Louisville) [18] was utilized for the detection of *P. gingivalis*, which was incubated with tissue sections (1:1,000 dilution) for 12 h at 4°C. Pre-immune rabbit IgG (CW0103, CWBIO, Beijing, China) and normal mouse IgG (CW0102, CWBIO, Beijing, China) was used as a negative control. As an additional control, sections were also incubated with 0.01 moL·L^−1^ phosphate buffered saline (PBS) only. Sections were counterstained with hematoxylin and visualized by light microscopy (Eclipse 80i, Nikon, Japan). According to the staining intensity and staining area of the cytoplasm and nuclei, four high-power microscopic fields (200 times) were randomly selected for observation in the tissue sections. Each tissue section was evaluated by two senior pathologists. Staining intensity and area were classified using a numerical scale. Staining intensity: zero, unstained; one point, buff; two points, claybank; three points, tan. Staining area (proportion of positive cells): zero, 0–10%; one point, 10–30%; two points, 30–60%; three points, >60%. IHC scoring was calculated by multiplying the staining intensity by staining area. A score of ≥2 was considered positive of staining with *P. gingivalis*.

### PCR Amplification

Tissues were suspended in 500 ml of sterile PBS, vortexed for 30 s and sonicated for 10 s. Proteinase K (2.5 mg/ml final concentration) was added and the samples were incubated overnight at 55°C, homogenized with a sterile disposable pestle and vortexed. DNA was extracted with a Tissue DNA Kit (D3396-01, OMEGA bio-tek, Georgia, America). All samples were stored at −80°C until further analysis. PCR for amplification of 16 S rDNA of *P. gingivalis* was performed in a total volume of 25 μL containing 2 mM of primers and 10 ng of template DNA. 16 S rDNA samples were amplified with 2xTaq Plus Master Mix (P211, Vazyme, Nanjing, China) as described previously [19] using *P. gingivalis* specific and universal 16 S rDNA primers (*P. gingivalis* 16 S rDNA primer sequences were: 5′AGG​CAG​CTT​GCC​ATA​CTG​CG3’ (forward) and 5′ ACT​GTT​AGC​AAC​TAC​CGA​TGT 3′ (reverse), and the PCR product size was 404 bp; the universal 16 S rDNA primer sequences were 5′GAT​TAG​ATA​CCC​TGG​TAG​TCC​AC3′ (forward) and 5′CCC​GGG​AAC​GTA​TTC​ACC​G3’ (reverse), and the PCR product size was 688 bp). The PCR cycling conditions were 30 cycles of denaturation at 94°C for 30 s, annealing at 65°C for 30 s with a decrease of 0.2°C per cycle, and extension at 72°C for 30 s.

### Statistical Analysis

All statistical analyses were performed with the SPSS statistical package, version 17.0 (SPSS Inc., Chicago, IL, USA). Correlations between the presence of *P. gingivalis* and clinicopathologic factors as well as the agreement between the two different methods of IHC and PCR were analyzed by chi-square tests as appropriate. The *kappa* statistic was used to assess interobserver variability, with a score of >0.75 indicating excellent agreement. Overall survival was estimated using the Kaplan-Meier method and the log-rank test was employed to compare survival time differences in overall survival. *P* values of <0.05 were considered statistically significant.

## Results

### Different Frequencies of *P.gingivalis* Detection in Cancerous Tissues from Oral-Digestive Tract Cancer Tissues

We conducted IHC to detect the positive rate of *P. gingivalis* in paraffin-embedded samples of clinical cancerous specimens from oral-digestive tract cancer tissues. We found that *P. gingivali*s was primarily immunolocalized to epithelial cell cytoplasm, but bacterial antigens were occasionally present in the nuclei, and the positive staining showed brown-yellow granules, as shown in Figure 1. *P. gingivalis* staining was positive in 60.00% (30/50) of samples from OSCC, 46.00% (23/50) of samples from ESCC, and 20.00% (6/30) of samples from GCA, while positive staining was found in only 6.67% (2/30) of GC, and 2.86% (1/35) of CRC, as shown in Table 1.

**FIGURE 1:** Immunohistochemical detection of *P. gingivalis* in oral **(A)**, esophagus **(C)**, cardia **(E)**, stomach **(G)** and colorectal **(I)** cancerous tissues and their corresponding negatively stained tissues **(B, D, F, H, J)**. Shown are high-magnification (400×) micrographs of the tissues.

**TABLE 1:** Frequency of presence of *P. gingivalis* in various cancer tissues.

Tissues	*n*	No.(%) of positive samples	
		IHC	PCR
Oral carcinoma	50	30 (60.00)	28 (56.00)
Esophagus cancer	50	23 (46.00)	21 (42.00)
Cardiac cancer	30	6 (20.00)	5 (16.67)
Gastric cancer	30	2 (6.67)	1 (3.33)
Colorectal cancer	35	1 (2.86)	1 (2.86)

To control for false positives cause by possible cross reaction of antibodies, the amount of *P. gingivalis* 16 S rDNA in surgical specimens of various types of cancer was assessed by PCR. We found that 56.00% (28/50) of OSCC samples, 42.00% (21/50) of ESCC samples, and 16.67% (5/30) of GCA tissues were positive for this microorganism. In addition, 3.33% (1/30) of GC tissues and 2.86% (1/35) of CRC tissues contained detectable levels of *P. gingivalis* DNA fragments.

### Comparison of Different Methods for the Detection of *P. gingivalis*

Subsequently, we compared the results of IHC and PCR for the presence of *P. gingivalis* in various cancers to determine the agreement between these two different methods. The data revealed that the percentage of tissues positively stained with anti-*P. gingivalis* in PCR positive tumors was significantly higher than that in the PCR negative tumors (91% vs. 8%; *P* < 0.0001). There were only five cases with IHC scores of lower than 2 that were PCR positive. In addition, we found 11 cases that were IHC positive and PCR negative (see Table 2). The sensitivity and specificity of IHC were 91% (51/56) and 92% (128/139), respectively. The concordance rate was 91.8% (*kappa* = 0.806; *P* < 0.001) between IHC and PCR. These findings showed that there was excellence concordance between IHC and PCR for the detection of *P. gingivalis*.

**TABLE 2:** Concordance between IHC and PCR of *P. gingivalis* in various cancerous tissues.

IHC	PCR		*Kappa* value^a^	*P*
	+	−		
+	51	11	0.806	<0.001
−	5	128		

^a^ Kappa value > 0.7 excellent; 0.4–0.7, good; <0.4, poor agreement.

### *Porphyromonas gingivalis* Detection Is Positively Correlated With the Clinicopathologic Characteristics of OSCC and ESCC

Since we had demonstrated an association between *P. gingivalis* detection and OSCC or ESCC, we next sought to determine if the presence of *P. gingivalis* is associated with the progression of those cancers. Pathological information from the OSCC and ESCC patients is presented in Table 3. No matter whether it was oral cancer or esophageal cancer, the presence of *P. gingivalis* was not significantly associated with age, gender, smoking or drinking history, or differentiation of the tumors, while the presence of *P. gingivalis* was positively related to lymph node metastasis and the clinical stages of OSCC and ESCC (*P* < 0.05). Positive PCR rates for *P. gingivalis* were 77.8% and 60% in the lymphatic metastasis tissues in OSCC and ESCC, which were significantly higher than those of nonmetastatic samples (43.8%, 24.0%; *P*< 0.05). Additionally, the detection rates of *P. gingivalis* were 45.9 and 30.3% in patients with early stage OSCC and ESCC, which were significantly lower than those in the late stage (84.6 and 64.7%), and the difference was statistically significant (*P*< 0.05). Taken together, these results revealed that *P. gingivalis* detection is positively correlated with severe lymph node metastasis and clinical stage of OSCC or ESCC, suggesting that *P. gingivalis* could be a novel etiologic agent and potential prognostic indicator of these important malignant diseases. Because the detection rate of *P. gingivalis* in cardia, stomach and colorectal cancer is too low and the small sample size too small (Table 1), these data were not analyzed.

**TABLE 3:** Association between the presence of *P. gingivalis* and the clinicopathologic features of OSCC and ESCC patients.

Pathology factors	*P. gingivalis* for OSCC		*χ* ^*2*^	*P*	*P. gingivalis* for ESCC		*χ* ^*2*^	*P*
	(−)	(+)			(−)	(+)		
Gender			0.487	0.485			1.676	0.196
Male	12 (40.0%)	18 (60.0%)			17 (51.5%)	16 (48.5%)		
Female	10 (50.0%)	10 (50.0%)			12 (70.6%)	5 (29.4%)		
Age			0.298	0.585			0.006	0.939
<60	7 (38.9%)	11 (61.1%)			8 (57.1%)	6 (42.9%)		
≥60	15 (46.9%)	17 (53.1%)			21 (58.3%)	15 (41.7%)		
Smoking			1.469	0.226			2.339	0.126
No	14 (51.9%)	13 (48.1%)			16 (69.6%)	7 (30.4%)		
Yes	8 (34.8%)	15 (65.2%)			13 (48.1%)	14 (51.9%)		
Drinking			2.131	0.144			0.911	0.340
No	14 (53.8%)	12 (46.2%)			15 (65.2%)	8 (34.8%)		
Yes	8 (33.3%)	16 (66.7%)			14 (51.9%)	13 (48.1%)		
Differentiation			1.404	0.496			4.260	0.119
Well	8 (57.1%)	6 (42.9%)			7 (63.6%)	4 (36.4%)		
Moderately	10 (40.0%)	15 (60.0%)			20 (64.5%)	11 (35.5%)		
Poorly	4 (36.4%)	7 (63.6%)			2 (25.0%)	6 (75.0%)		
Lymph node metastasis			5.414	**0.020**			6.650	**0.010**
Yes	4 (22.2%)	14 (77.8%)			10 (40.0%)	15 (60.0%)		
No	18 (56.3%)	14 (43.8%)			19 (76.0%)	6 (24.0%)		
Clinical stage			5.838	**0.016**			5.451	**0.020**
I + II	20 (54.1%)	17 (45.9%)			23 (69.7%)	10 (30.3%)		
III + IV	2 (15.4%)	11 (84.6%)			6 (35.3%)	11 (64.7%)		

Bold text highlights statistically significant findings.

### *Porphyromonas gingivalis* Detection is Negatively Correlated with the Overall Survive Rate of OSCC and ESCC

To assess the potential consequences of *P. gingivalis* detection in OSCC and ESCC patients, we next compared the overall cumulative survival rate in OSCC and ESCC patients with and without *P. gingivalis* detection (see Table 4). We found that the overall survival rate was significantly higher in the *P. gingivalis* undetected group (86%) than that in the detected group (57%) with OSCC. The median survival time (SMT) was 39 months in the *P. gingivalis* detected group, significantly lower than that of the *P. gingivalis* undetected group. Similar results were found for the ESCC *P. gingivalis* undetected group (50%) and *P. gingivalis* detected group (14%). The MST for patients with *P. gingivalis* detection was 40 months, significantly lower than that of the *P. gingivalis* undetected group (64 months). Furthermore, Kaplan–Meier analysis showed that *P. gingivalis* presence was significant for overall survival both for OSCC (*n* = 50, *χ* ^*2*^ = 5.929, *P* = 0.015) (Figure 2A) and ESCC (*n* = 50, *χ* ^2^ = 4.086, *P* = 0.043) (Figure 2B). These results indicated that the prognoses of *P. gingivalis* detected groups of OSCC and ESCC patients was poor.

**TABLE 4:** The overall survival rate and medians survival time (months) of OSCC and ESCC patients with the presence of *P. gingivalis*.

Tissues	Case (*N* = 50)	OS(%)	MST (months)	*χ* ^*2*^	*P*
OSCC				5.929	0.015
*P. gingivalis* (+)	28	57	39		
*P. gingivalis* (−)	21	86	–		
ESCC				4.086	0.043
*P. gingivalis* (+)	21	14	40		
*P. gingivalis* (−)	29	50	64		

**FIGURE 2:** Kaplan–Meier survival analysis of the relationship between the presence of *P. gingivalis* and the overall survival rate of OSCC and ESCC patients. Higher expression of the *P. gingivalis* whole cell antigen was positively related with poorer overall survival of both OSCC **(A)** and ESCC **(B)** patients. The *P* value is 0.015 **(A)** and 0.043 **(B)** respectively.

## Discussion

The correlation between bacterial infection and the development of cancer has been a focus of cancer research in recent years. *P. gingivalis* is a Gram-negative anaerobe living in oral gingival epithelial cells. As one of the three major pathogenic bacteria of the “red complex” in the oral cavity [20], *P. gingivalis* is a key bacterium of the overall oral microecological balance. The special anatomical structure and environment of the oral cavity endow *P. gingivalis* with important pathophysiological significance, and extensive blood-borne invasion can promote *P. gingivalis* to participate in systemic diseases [9]. In recent years, many studies have shown that *P. gingivalis* are positively correlated with clinical risks of systemic diseases such as Alzheimer's disease, coronary atherosclerosis, respiratory tract infections, and osteoporosis [21–23]. *P. gingivalis* has also been proven to be an the important etiological agent of head and neck squamous cell carcinoma and lung cancer and an important pathogenic bacterium that mediates long-term chronic infection [24, 25].

Previous studies have confirmed that there is a close relationship between oral microorganisms and the occurrence and development of OSCC [26, 27]. Increasingly studies have shown that *P. gingivalis*, as the dominant bacterium in periodontitis, is correlated with OSCC. In 2011, Katz et al. [12] found that *P. gingivalis* expression was much higher in OSCC tissue than normal tissue by comparing samples from 10 cases of OSCC and 5 healthy subjects using IHC analysis; they also examined the symbiotic bacterium *Streptococcus gordonii* as a reference and found no any difference. Although the sample size of that study was small, this was the first report of a significant positive correlation between *P. gingivalis* detection and the occurrence of OSCC. In addition, Chang et al. [28] found that the detection rate of *P. gingivalis* in gingival squamous cell carcinoma was about 45%, that of tongue squamous cell carcinoma was about 40%, and that of normal gingivalis tissue was about 20% by analyzing the samples from patients with OSCC in China; the difference between OSCC and normal tissue was statistically significant. Furthermore, the authors’ [20] bibliographic research was carried out selecting articles published until 2020, Seventeen articles, 14 *in vitro* and three in animal models were selected. According to authors, *P. gingivalis* could play an important role in OSCC development and could be involved in three different stages: epithelial–mesenchymal transition of malignant cells, neoplastic proliferation, and tumor invasion [29]. In the present study, DNA fragments from the cancer tissues of the oral-digestive tract showed that *P. gingivalis,* known for its strong virulence, preferentially infects OSCC, and the detection rate was 56.00%. *P. gingivalis* detection was related to lymph node metastasis, clinical stage, and prognosis, suggesting that *P. gingivalis* detection is involved in the development and metastasis of oral cancer, which is consistent with the above reports. As a multi-pathogenic factor of OSCC, there is no clear evidence to prove a causal relationship between *P. gingivalis* and OSCC so far. The role of *P. gingivalis* in the pathogenesis of OSCC remains unclear, and it is possible that it is only a synergistic pathogenic factor of OSCC. More large-scale studies are needed to confirm the exact relationship and underlying mechanism between *P. gingivalis* and OSCC.

*Porphyromonas gingivalis* is found in the saliva of healthy subjects and patients with ESCC [30]. Due to the continuity of the physiological structure between the esophagus and the oral cavity, ESCC is more susceptible to oral flora than other parts of the digestive system [31, 32]. Therefore, *P. gingivalis* may be transferred to the esophagus along with food or saliva. In 2016, our team first found that *P. gingivalis* is a high risk factor of esophageal cancer [14]. In 2017, we confirmed that *P. gingivalis* widely colonizes esophageal cancer and precancerous tissue, that the abundance is lower in adjacent and normal mucosal tissues, and that its content is very low or absent in cardia and gastric cancer; we attributed this difference to the low tolerance of *P. gingivalis* to an acidic environment [13]. In 2020, we investigated the molecular mechanisms driving aggressive progression of ESCC by *P. gingivalis*. Intracellular invasion of *P. gingivalis* potentiated proliferation, migration, invasion, and metastasis abilities of ESCC cells via transforming growth factor-β (TGFβ)-dependent Drosophila mothers against decapentaplegic homologs (Smads)/Yes-associated protein (YAP)/Transcriptional coactivator with PDZbinding motif (TAZ) activation [33]. In addition, Chen et al. [34] discovered that the presence of *P. gingivalis* was associated with advanced clinical stages and a poor prognosis. Our current study also found that *P. gingivalis* was present in esophageal epithelial cells of ESCC patients with an detection rate of 42.00%, and that was related to the severity and prognosis of ESCC. These findings indicate that *P. gingivalis* may be used for ESCC screening and prognosis monitoring, and it is conducive to the early detection of ESCC. Hence, further studies to determine if *P. gingivalis* infection promotes the initiation and progression of ESCC are required.

There are few studies about *P. gingivalis* and GCA or GC. In a cross-sectional study, Salazar et al. [35] detected the DNA expression levels of several periodontal pathogens including *P. gingivalis* in dental plaques and saliva samples from 37 cases of chronic atrophic gastritis, intestinal metaplasia, and atypical hyperplasia of patients with periodontitis using real-time quantitative PCR; they found that the colonization of three kinds of periodontal pathogens, *P. gingivalis*, *Treponema denticola,* and *Tannerella forsythia,* in dental plaques increased the risk of precancerous lesions of GC. In the present study, the detection rates of *P. gingivalis* in GCA and GC were 16.67 and 3.33%, respectively, which is consistent with previous reports from our team. Yuan et al. [13] discovered that *P. gingivalis* cannot survive in environments with high acidity and decreases with increasing acid levels and bacterial flora formation, thereby causing low infection of *P. gingivalis* in the stomach and cardia. The relationship between *P. gingivalis* and GC requires further study. In recent years, the role of intestinal microbiota changes and the formation of the tumor microenvironment in the occurrence and development of CRC has attracted increasing attention [36, 37]. Although studies have shown that *Fusobacterium nucleatum* is closely related to the occurrence and development of CRC, due to the complexity of intestinal flora, the development of CRC may not only be related to this kind of bacterium [6]. In this study, *P. gingivalis* detection was also found in CRC tissues, but the detection rate was low (2.86%). In a case control study, Wu et al. [38] analyzed and compared the intestinal microbiota between CRC patients and tumour-free subjects utilizing next-generation sequencing technology (16 S rRNA pyrosequencing analysis) in fecal samples, and they found that *Porphyromonas* was much higher in fecal samples of colon cancer patients than in healthy subjects. In another study, 16 S rRNA gene sequencing in fecal samples revealed reduced overall diversity of the intestinal microbiota, with elevated numbers of *Fusobacterium* spp. and *Porphyromonas* spp. and reduced abundance of *Clostridium* spp., between fecal samples from CRC patients and controls [39]. In 2017, increased abundance of periodontal pathogens such as *Fusobacterium, Oscillibacter, Peptostreptococcus, Porphyromonas, Roseburia, and Ruminococcus* were also observed in fecal samples from patients with CRC [40, 41]. The above studies showed that *Porphyromonas* was only found in the feces of patients with CRC, and not found in cancer tissues. The present study is the first to discover *P. gingivalis* detection in CRC tissues.

## Conclusion

In summary, in this study we found frequent detection of *P. gingivalis* in OSCC, but it was much less frequent in GCA and was absent from GC and CRC. These findings, though require further confirmation from large independent studies, seem to support the notion that *P. gingivalis* detection shows a decreasing distribution pattern in oral-digestive tract tumors. *P. gingivalis* may get into the esophagus and cardia through the oral cavity, and almost disappear in the stomach and colorectal tract due to gastric acid. In addition, *P. gingivalis* could plays an important role in promoting the occurrence and development of OSCC and ESCC, and may be an important risk factor. As a consequence, *P. gingivalis* may be used as a biomarker to evaluate the malignant degree and prognosis of OSCC and ESCC. The prevention and treatment of *P. gingivalis* infection may improve therapy and prognosis, but this needs to be supported by further basic and clinical research evidence.

## Availability of Data and Material

The data that support the findings of this study are available from the First Affiliated Hospital of Henan University of Science and Technology. Restrictions apply to the availability of these data, which were used under license for this study. Data are available from the authors with the permission of the First Affiliated Hospital of Henan University of Science and Technology.

## Data Availability

The original contributions presented in the study are included in the article/Supplementary Material, further inquiries can be directed to the corresponding authors.
